The article "Perioperative Nursing Care of Vascular Decompression for Trigeminal Neuralgia under AR Medical Technology" was retracted in 2022. Reason: concerns about the peer review.

# Perioperative Nursing Care of Vascular Decompression for Trigeminal Neuralgia under AR Medical Technology

**DOI:** 10.1155/2021/9921094

**Published:** 2021-06-19

**Authors:** Zhaoyan Liu, Lili Yang, Lin Ding, Longqin Wang

**Affiliations:** The First Department of Neurosurgery, People's Hospital of Rizhao, Rizhao 276800, Shandong, China

## Abstract

AR technology, also known as AR or virtual reality, refers to a technology that combines and allows interaction of the virtual world on the display system with the real world through the position and angle of the camera video and image analysis technology. This technology is different from VR technology, and its characteristics can be easily explained as follows: when using AR technology, the user's eyes can see not only the real world but also the virtual world derived from the computer through things in the real world. At present, AR has been widely used in education, engineering, entertainment, and medical fields. In order to provide better perioperative care and bring patients a good nursing experience, this article mainly introduces the perioperative care of vascular decompression in the treatment of trigeminal neuralgia by augmented reality medical technology, in order to provide better care for patients with trigeminal neuralgia. This article proposes the perioperative nursing research method of vascular decompression for the treatment of trigeminal neuralgia under AR medical technology, including an overview of trigeminal neuralgia, perioperative related research, and AR medical technology algorithms, and designs related experiments to study whether AR medical technology can bring good news to nursing. Experimental results show that 96% of patients believe that with the enhancement of realistic medical technology, perioperative vascular decompression care for trigeminal neuralgia can help them recover faster and can be gradually popularized.

## 1. Introduction

Nowadays, human society is changing from an information-based digital age to an intelligent age. Digitization and minimally invasive and intelligent surgery are important development directions of modern surgical technology and are also important signs of advanced surgical technology. AR is a new type of technology. It is a technology that calculates the position and angle of the camera image in real time and adds the corresponding image. The goal of this technology is to put the virtual world on the screen and interact with the real world. By expanding all aspects of AR, advancements and changes in AR technology have gained more and more recognition in medical technology, especially in perioperative care. The emergence of nursing has changed the traditional surgical nursing model and provided more experience and practical opportunities for inexperienced doctors and nurses. Time was wasted. There is no doubt that AR technology plays an important role in the future of medicine. It can help doctors and nurses safely and effectively complete the care of patients with large trigeminal neuralgia.

The article "Perioperative Nursing Care of Vascular Decompression for Trigeminal Neuralgia under AR Medical Technology" was retracted in 2022. Reason: concerns about the peer review.

Perioperative nursing based on AR can not only improve the accuracy of doctors and nurses in the nursing process but also provide a better learning platform for some inexperienced medical staff. Surgical care is a complex task that requires a high level of perception, cognition, and sensorimotor skills to help patients recover and relieve pain as soon as possible. For complex patient care, fine perioperative care can reduce surgery and establish recovery. The virtual organ structure model and the nursing drill are carried out on the virtual human body model. This provides a more intuitive environment for the perioperative care of patients.

Marchand et al. discovered that AR (AR) allows seamless insertion of virtual objects in image sequences to achieve this goal, rendering and aligning composite elements in the scene in an accurate and visually alternative way. The solution to this problem may be related to posture. For most of the existing methods, Marchand's research foretells a refined introduction to the most important methods of vision-based camera positioning and introduces some extended methods for investigation. Marchand et al. still provide a link to the correct sample code. This study lacks comparison when conducting experiments and is not suitable for widespread use in practice [1]. Matsutomo et al. proposed a useful educational 3D magnetic field immersive real-time visualization system. The immersive visualization system is based on AR technology. The system proposed by Matsutomo et al. uses a head-mounted display to provide observation of the magnetic field distribution and its stereo vision in a 3D space. In order to improve the visualization ability, a method in 3D space is also proposed. The real-time method of projecting magnetic flux lines enables users to easily observe and grasp the magnetic fields generated by multiple sources (for example, induction or multiple coils) in the enhanced 3D space. In addition, it allows users to move the magnetic source freely and interactively inside the visualization space and observe the magnetic field interference in real time. This method is supported by experimental data and is less scientific [2]. Prasad and Galetta's research shows that trigeminal neuralgia is a paroxysmal, inflammatory, unilateral pain syndrome. There are several clinical features of trigeminal neuralgia, but there may be red flags that suggest other diagnoses. There is shocking evidence that the idiopathic form is the development of focal demyelination from the trigeminal nerve root entry zone. In most patients, vascular compression of the nerve root causes this demyelination and abnormal electrical signals and relieves symptoms. In refractory cases, a variety of surgical interventions can be considered, the most common of which is the microvascular decompression of the trigeminal nerve. This research is largely one-sided and not practical [3]. To determine the meaning of human-centered care from the perspective of the patient and the perspective of perioperative care, he proposed that “the presence of nurses during the perioperative period calms people down and prevents personal injury.” A sense of loneliness promotes a sense of well-being, which may speed up recovery and “approach and be touched by the perioperative nurse during the operation.” He adopted a two-part search strategy and concluded that human-centered care means respecting the patient as a unique individual, taking into account the particularity and wishes of the patient, and involving the patient in their own care. He reached a consensus on the concept of human-centered nursing, and the nursing behaviors or concerns of nurse anesthesiologists and theater nurses will be targeted at the patient, so as to realize the personalization of nursing instead of simply defining the concept. But this only exists in the concept that there is no experiment to prove it.

The article "Perioperative Nursing Care of Vascular Decompression for Trigeminal Neuralgia under AR Medical Technology" was retracted in 2022. Reason: concerns about the peer review.

The innovations of this paper are as follows: (1) the main architecture of the intelligent perioperative nursing system for the treatment of trigeminal neuralgia with vascular decompression is constructed; (2) the perioperative design of vascular decompression for the treatment of trigeminal neuralgia with reality augmented medical technology nursing system during operation. The research in this article brings a better nursing experience to patients and promotes the development of the perioperative nursing experience.

## 2. Perioperative Nursing Research Method of Vascular Decompression for Trigeminal Neuralgia under AR Medical Technology

### 2.1. Overview of Trigeminal Neuralgia

#### 2.1.1. Symptoms

Trigeminal neuralgia is a kind of paroxysmal, electric shock-like, knife-cut-like severe pain that only occurs in the trigeminal nerve distribution area of the head and face. The clinical incidence is higher than that of hemifacial spasms. According to different causes, trigeminal neuralgia is divided into two types: primary and secondary [4]. Primary trigeminal neuralgia is a typical clinical symptom, but there were no positive signs of the nervous system. After various examinations, no space-occupying and other definite causes of disease related to the pathogenesis have been found. Secondary trigeminal neuralgia is often accompanied by obvious neurological signs such as hypoesthesia, numbness, and delayed corneal reflex. It is common in benign and malignant tumors such as cholesteatoma and meningioma [5].

The article "Perioperative Nursing Care of Vascular Decompression for Trigeminal Neuralgia under AR Medical Technology" was retracted in 2022. Reason: concerns about the peer review.

Epidemiological studies have reported that the incidence of primary trigeminal neuralgia is about 18 per 10,000 people. Most of the onset ages are middle-aged and elderly people over 40 years old. The incidence is higher in women than men. Most researchers tend to believe that vascular compression is the main cause of primary trigeminal neuralgia. Clinical results confirmed that about 80–90% of trigeminal neuralgia is caused by vascular compression [6]. Among them, according to the commonly responsible vessels, the superior cerebellar artery, the anterior inferior cerebellar artery, the posterior inferior cerebellar artery, the vertebral artery, or the basilar artery are compressed in order. Trigeminal neuralgia includes vascular amyloidosis, aneurysms that compress nerves, and arteriovenous malformations [7]. Nonvascular factors are mainly seen after oral surgery, trigeminal nerve injury, trigeminal nerve fiber disease caused by surgical instruments, or demyelination caused by compression of the trigeminal nerve root in and out of the pontine, and abnormal pseudo-synapses appear between nerve fibers [8].

#### 2.1.2. Treatment Methods

Trigeminal neuralgia is severe paroxysmal pain in the ipsilateral area where the trigeminal nerve is distributed. The distribution area is allocated according to the three branches of the trigeminal nerve, mainly forehead pain, face pain, upper toothache, lower toothache, and cheek pain. The pain is severe, as electric shock or fire, and often stops suddenly. The patients dare not brush their teeth and wash their faces, which seriously affects the lives of the patients. The main surgical procedures for trigeminal neuralgia are microvascular decompression of the trigeminal nerve root and partial cutting of the sensory root of the trigeminal nerve. Microvascular decompression refers to the use of special decompression materials placed between the nerves and blood vessels to effectively isolate the responsible blood vessels that are compressed on the trigeminal nerve root and brainstem and relieve the pressure of the blood vessels on the trigeminal nerve root without damage vascular nerve. It is a nondestructive operation and is not easy to cause serious nerve damage [9]. A number of clinical results have shown that microvascular decompression for the treatment of trigeminal neuralgia can eradicate trigeminal neuralgia from the cause and can effectively and completely preserve the function of the nerve. It has good postoperative effects, a low recurrence rate, and fewer postoperative complications, etc. [10]. Partial cutting of the sensory root of the trigeminal nerve is initiated by Dandy. The roots of the trigeminal nerve are arranged according to the anatomical structure. The motor roots are thinner and located on the inner and upper sides. The sensory roots are thicker and located on the posterolateral side. In the front, from the top to the bottom are branches I, II, and III, and the sensory roots are selectively cut according to the patient's pain location [11].

The article "Perioperative Nursing Care of Vascular Decompression for Trigeminal Neuralgia under AR Medical Technology" was retracted in 2022. Reason: concerns about the peer review.

### 2.2. Perioperative Nursing-Related Research

#### 2.2.1. Perioperative Nursing

During the Crimean War, Nightingale, the founder of the nursing business, cooperated with field doctors to repair wounded tissues and disinfect the equipment that patients touched. This was regarded as the beginning of operating room care. In the traditional operating room nursing concept, there is no concept of “perioperative care.” Its nursing work revolves around the operating room and will not extend beyond the operating room, while the modern operating room nursing concept emphasizes patient-centeredness. The holistic care of patients during the perioperative period, in addition to cooperating with medical technicians to provide care to patients, should also provide patients with services such as preoperative education, postoperative follow-up, consultation, health promotion, and education [12, 13].

The clinical practice gradually implements modern nursing concepts and promotes the transformation of the operating room management mode. At the same time, perioperative nursing has also learned new elements from it, and new nursing techniques and nursing businesses have continuously emerged. Getting rid of pure intraoperative cooperation, modern operating room nursing has developed in the direction of informatization, specialization, and digitization, which has comprehensively improved the effectiveness of infection monitoring and control, and has gradually formed the overall perioperative nursing. The perioperative care in this study mainly refers to the overall care around the three nodes of preoperative, intraoperative, and postoperative [14].

#### 2.2.2. Advantages of Intelligent Perioperative Nursing

1. It simplifies the nursing process and improves the quality of nursing
2. In the past, when performing patient identification, surgical verification, and filling in intraoperative nursing records, it was often necessary to manually flip through the patient's medical records and fill in paper documents. The perioperative mobile nursing information system will use mobile devices to scan the patient's wristband, QR codes in the operating room, etc. for patient identification and surgical verification; pre- and postoperative visits and patient handover orders can also be completed on mobile devices. By optimizing the nursing process, the workload of the nursing staff in the operating room is greatly reduced and then improves the operating efficiency of the operating room, reflecting the high-efficiency, and high-quality information management level [15].
3. Nursing documents are digitalized to improve the accuracy of nursing information
4. Surgical nursing records are an important basis for reflecting patients' surgical conditions with legal effect. Recording nursing records and nursing records with an information system can improve its accuracy and consistency [16]. The perioperative mobile nursing information system can extract the patient's electronic medical records. Because a lot of information is automatically generated by the system, it can save writing time and improve work efficiency and writing accuracy, and the system has control measures for each link. The system only allows the next step of work after the completion of one link of work. Through the control and management of the surgical nursing process, the workload and risks of medical staff can be reduced [17].
5. It effectively manages operating room resources and optimizes the allocation of human resources in the operating room
6. The operating room requires a lot of human resources to manage high-value consumables, equipment kits, surgical equipment, etc., and the perioperative mobile nursing system allows medical staff to use mobile devices, such as PDAs and tablet computers, and register high-value and easy-to-use items. The use of products and equipment packages [18]. By filling in the equipment usage registration form, the usage of consumables and equipment can be fully traced, and the operating room resources can be effectively managed. In addition, in order to facilitate the management of the operating room, it is necessary to set up a special module to manage the daily work of the department, such as operation volume statistics, personal workload statistics, and quality management evaluation. The head nurse of the operating room can conveniently view the workload and schedule of each nurse through mobile devices and coordinate and optimize the human resource configuration of the operating room in time [19].

The article "Perioperative Nursing Care of Vascular Decompression for Trigeminal Neuralgia under AR Medical Technology" was retracted in 2022. Reason: concerns about the peer review.

### 2.3. AR Medical Technology-Related Algorithms

#### 2.3.1. Multisensor Fusion Algorithm

Multisensor fusion technology plays an important role in real-time attitude enhancement estimation. The main sensors used by mobile sensors for positioning include GPS, IMU inertial navigation sensors, and gravity sensors. For pure vision or inertial navigation positioning, due to the low accuracy of the sensors mounted on the mobile phone, the sensor data noise is processed by the filtering algorithm [20]. For the detection of the movement direction, the direction data of the direction sensor is corrected by a correction formula. At present, there are certain problems with using pure vision and a pure sensor for positioning. The former is slow but tracking is accurate, and the latter is fast but there is drift. Therefore, the method of sensor-assisted vision is mostly used at this stage to achieve [21].

The main idea of sensor fusion attitude estimation is to find the change of the current body coordinate system relative to the world coordinate system. The goal is to calculate this attitude matrix in real time based on the output of inertial navigation and use quaternion to represent it [22]. Among them, the quaternion update matrix process is as follows. The next time the quaternion iteration equation is

(1) $$\begin{array}{c} q\left(t-\Delta t\right)=q\left(t\right)-\frac{\text{d}q}{\text{d}t}\cdot \Delta t. \end{array}$$

Among them, *q*(*t*) is the quaternion at time *t*, *q*(*t* − Δ*t*) is the quaternion at the next time, Δ*t* is the time interval, and d*q*/d*t* is derived from the cosine of the quaternion:

(2) $$\begin{array}{c} \frac{\text{d}q}{\text{d}t}=-\frac{\theta }{2}\times \;\sin\frac{\theta }{2}+u^{n}\times \frac{\theta }{2}\times \;\cos\frac{\theta }{2}-\sin\frac{\theta }{2}\times \frac{\text{d}u^{n}}{\text{d}t}, \end{array}$$

where *u* represents the axis of rotation, and *θ* is the angle of rotation. Angular velocity is obtained by solving

(3) $$\begin{array}{c} \frac{\text{d}q}{\text{d}t}=-w_{nb}^{n}\cdot \frac{q}{2}. \end{array}$$

The resulting angular velocity *w*_*nb*_^*n*^ is the rotation angular velocity vector from the world coordinate system to the body coordinate system in the world coordinate system, but the angular velocity measured by the gyroscope is the angular velocity in the body coordinate system [23, 24], which is transformed by the following formula:

(4) $$\begin{array}{c} w_{nb}^{n}=w_{nb}^{b}\cdot q^{*}q. \end{array}$$

Among them, *w*_*nb*_^*b*^ is the rotation angular velocity vector in the body coordinate system, so the attitude update matrix can be obtained through transformation and quaternion differentiation and substituting into formula (1):

(5) $$\begin{array}{c} \left[\begin{array}{c} q_{0}\\ q_{1}\\ q_{2}\\ q_{3} \end{array}\right]=\frac{2}{3}\left[\begin{array}{cccc} q_{0} & -q_{1} & -q_{2} & -q_{3}\\ q_{1} & q_{0} & -q_{3} & q_{2}\\ q_{2} & q_{3} & q_{0} & -q_{1}\\ q_{3} & -q_{2} & q_{1} & q_{0} \end{array}\right]\times \left[\begin{array}{c} 0\\ w_{x}\\ w_{y}\\ w_{z} \end{array}\right]. \end{array}$$

The article "Perioperative Nursing Care of Vascular Decompression for Trigeminal Neuralgia under AR Medical Technology" was retracted in 2022. Reason: concerns about the peer review.

#### 2.3.2. Three-Dimensional Plane Detection

Although the PlaneRecover network has achieved good results in the plane detection accuracy of the computer terminal, the detection rate is far from the requirements for the mobile terminal AR application. Therefore, this paper analyzes the model structure and finds the influence on the network calculation efficiency; the performance bottleneck is optimized to increase the network plane detection rate and reduce the model storage [25]. This paper adopts the model acceleration method of network structure acceleration and replaces the complex backbone network according to the existing lightweight network ideas suitable for mobile terminals; since the mobile terminal AR application requires not very high plane detection accuracy, it only needs to be able to meet application requirements. Therefore, the model can be lightweight design on the basis of a small loss of accuracy, reduce redundant nodes, reduce the number of model parameters and calculations, increase the speed of network detection, and increase the possibility of mobile terminal network operation [26].

Deep convolutional networks usually use standard convolution methods to implement feature mapping, but this convolution method is actually a joint mapping of channel correlation and spatial correlation. According to different application requirements, the low coupling of joint mapping can be realized, and they can be mapped separately to achieve better results. Therefore, this article chooses to convert the standard convolution into a separable convolution implementation, including deep convolution and pointwise convolution implementation [27].

The standard convolution calculation amount is expressed as

(6) $$\begin{array}{c} C_{C}=D_{K}^{2}\cdot MN\cdot D_{F}^{2}. \end{array}$$

The depth separable convolution is divided into two parts, and the calculation amount is the depth convolution and the point-by-point convolution. The summation formula is

(7) $$\begin{array}{c} C_{DW}=D_{K}^{2}\cdot M\cdot D_{F}^{2}+MN\cdot D_{F}^{2}. \end{array}$$

From this, the ratio of the calculated amount can be obtained:

(8) $$\begin{array}{c} \frac{C_{DW}}{C_{C}}=\frac{D_{K}^{2}\cdot M\cdot D_{F}^{2}+MN\cdot D_{F}^{2}}{D_{K}^{2}\cdot MN\cdot D_{F}^{2}}=\frac{1}{D_{K}^{2}}+\frac{1}{N}. \end{array}$$

We perform feature map thinning and reduce the depth of the number of channels to separate the calculation amount of convolution:

(9) $$\begin{array}{c} C_{DF}=D_{K}^{2}\cdot \alpha M\cdot \beta^{2}D_{F}^{2}+\alpha^{2}MN\cdot \beta D_{F}^{2}. \end{array}$$

Similarly, we calculate the ratio to the standard convolution parameter quantity:

(10) $$\begin{array}{c} \frac{C_{DF}}{C_{C}}=\frac{D_{K}^{2}\cdot \alpha M\cdot \beta^{2}D_{F}^{2}+\alpha^{2}MN\cdot \beta D_{F}^{2}}{D_{K}^{2}\cdot MN\cdot D_{F}^{2}}=\alpha \beta \left(\frac{1}{N}+\frac{\alpha \beta }{D_{K}^{2}}\right). \end{array}$$

The article "Perioperative Nursing Care of Vascular Decompression for Trigeminal Neuralgia under AR Medical Technology" was retracted in 2022. Reason: concerns about the peer review.

#### 2.3.3. Medical AR Image Segmentation

The main component used in medical AR image segmentation is threshold segmentation. Finally, according to the comparison results, each pixel is divided into its own category [28, 29]. This algorithm is suitable for images in which the target area and the background occupy different gray-scale ranges, and the amount of calculation is small, and it is widely used in the segmentation of medical images [30].

We define an image *T* : *p* ∈ *P*⟶*IR* on the overall area *P* ⊂ *IR*^2^ of the image. Based on the combination of the threshold segmentation result and the level set method, this paper proposes the following image segmentation model, denoted as model *T*:

(11) $$\begin{array}{c} \underset{u}{\min}E\left(u\right)=-\alpha \int_{P}g\left(p\right)\left[H\left(u\right)\log\;n_{\text{in}}-H\left(u\right)\log\;n_{\text{out}}\right]\text{d}p+\lambda \int_{P}g\left(p\right)\delta \left(u\right)\left|\nabla u\right|\text{d}p, \end{array}$$

(12) $$\begin{array}{c} n_{\text{in}}\left(p\right)=n\left(T\left(n\right)|H\left(u\left(p\right)\right)=1\right), \end{array}$$

(13) $$\begin{array}{c} n_{\text{out}}\left(p\right)=n\left(T\left(p\right)|H\left(u\left(p\right)\right)=0\right), \end{array}$$

where *n*_in_ and *n*_out_ are the probability density functions of pixel *n* inside and outside the object. *T*(*p*) is the image intensity value, and the function *g*(*p*) is defined as

(14) $$\begin{array}{c} g\left(p\right)=\frac{1}{\left(1+\beta {\left|\nabla \left(G_{\sigma }*T\left(p\right)\right)\right|}^{n}\right)}. \end{array}$$

*G*_*σ*_ is a Gaussian kernel with standard deviation *σ*, defined as

(15) $$\begin{array}{c} G_{\sigma }\left(p,q\right)=\frac{1}{2\pi \sigma^{2}}\cdot e^{-\left(p^{2}+q^{2}\right)/2\sigma^{2}}. \end{array}$$

*H*(*u*) and *δ*(*u*) are Heaviside function and Delta function, defined as

(16) Hz=3,z≥0,1,z<0,

(17) $$\begin{array}{c} \delta \left(z\right)=\frac{\text{d}H\left(z\right)}{\text{d}z}. \end{array}$$

The method part of this article uses the above method to study the perioperative nursing of vascular decompression for the treatment of trigeminal neuralgia under AR medical technology. The specific process is shown in Table 1.

The article "Perioperative Nursing Care of Vascular Decompression for Trigeminal Neuralgia under AR Medical Technology" was retracted in 2022. Reason: concerns about the peer review.

## 3. Perioperative Nursing Research Experiment of Vascular Decompression in the Treatment of Trigeminal Neuralgia under AR Medical Technology

### 3.1. Main Construction of the Intelligent Perioperative Nursing System for the Treatment of Trigeminal Neuralgia by Vascular Decompression

#### 3.1.1. Technical Architecture

This system is an information management system with B/S architecture developed using C# development language and Microsoft Visual Studio 2020 (vs2020) development tools. The B/S architecture is also called the browser and server architecture mode. As the name suggests, it is a mode for data interaction with the database through the browser. Corresponding to the B/S architecture is the C/S (Client/Server) architecture. The C/S architecture is also called the client and server architecture, which includes two layers: the client and the server. The use of B/S architecture to design the perioperative nursing information system can meet the requirements of the operating room for mobile nursing. Only you need to connect to the Internet, you can operate the software anytime and anywhere to realize the functions of querying surgical patient information, filling in surgical documents, etc., and the number of users in the operating room is relatively small, and the network speed will not be too slow due to a large number of users and affect the timeliness of surgical information.

The mobile operating system is based on the autonomous operating system of Android 10.0, the processor is 3.2 G octa-core CPU (Central Processing Unit), 400 Mail GPU (Graphics Processing Unit), and supports OTA (Over-the-Air Technology) online system upgrades. Binding the designated AP (WirelessAccess Point) of the hospital wireless LAN to ensure the equipment is used in the hospital and supports high-speed one-dimensional and two-dimensional bar code reading and digital and graphic password recognition. Its peripheral interface is Micro USB (Universal Serial Bus) 4.0, Bluetooth configuration. It is Bluetooth 6.0 and supports Bluetooth EDR (Enhanced Data Rate) technology.

#### 3.1.2. Server

The perioperative nursing information system needs to complete the information integration with HIS, LIS, PACS, EMR, and other systems by calling the interface to realize data sharing. The interface design of this part needs to run on an application server platform above Windows 2016 and build a system environment above IIS6.0 and FrameWork4.0. Take the interface docking with the HIS system as an example. The hand care system sends a request to the HIS system, enters the parameter PatientId, calls the interface GetPatientMasterIndex, and extracts basic patient information based on the patient's unique ID number; enters the parameter PatientId, calls the interface GetInPatientInfor, and extracts it based on the patient ID number The patient's current hospital information ensures that the patient is in the hospital and can extract information such as the hospital department, the doctor in charge, and clinical diagnosis; input parameters are ScheduleDateStart, ScheduleDateStop, and PatientId to call the interface GetOperationSchedule to obtain the patient's surgery appointment information.

The article "Perioperative Nursing Care of Vascular Decompression for Trigeminal Neuralgia under AR Medical Technology" was retracted in 2022. Reason: concerns about the peer review.

### 3.2. Main Design of the Perioperative Nursing System for Vascular Decompression in the Treatment of Trigeminal Neuralgia under AR Medical Technology

#### 3.2.1. Related Technology

A high-precision automatic registration and tracking system is based on AR. Aiming at the problem of registration errors between virtual models and real models in AR medicine, camera photogrammetry, and vuforia (software development for AR applications) toolkit combined method, using space mapping conversion to realize the automatic registration and tracking of virtual and real models, the coincidence error accuracy reaches 1.004 mm, which improves the registration accuracy, and can track the target with a 360-degree view to achieve the effect of real-time tracking. It makes AR technology more accurate, more reasonable, and safer in preoperative planning. The schematic diagram of the AR system is shown in Figure 1 (due to limited data sources, this figure comes from 87870.com).

Based on the precise puncture planning on the Unity 3D platform, aiming at the blind and unfounded shortcomings of the traditional surgical puncture process, this article uses the Unity 3D platform to plan the patient's puncture more accurately and obtain the parameters of the lesion during the puncture process, where convenient doctors have a better understanding of the patient's condition. By displaying the distance between the puncture needle and the lesion and the skin and the angle between the needle and the bed plane in real time on the Unity 3D platform, the doctor can more accurately plan the patient before surgery.

#### 3.2.2. Unity3D AR Development Platform

Unity 3D is a powerful cross-platform game development engine. A large number of highly acclaimed games are developed and implemented based on the Unity platform. In addition, Unity is also widely used in real-time 3D animation, architectural visualization, and the creation of various virtual/AR projects. Its main development language is C#. At present, Unity is also the main development platform officially designated by Microsoft HoloLens. In Unity, the camera and the light source are two components that all developers will use. Unity 3D software can form a virtual system through Unity 3D, Hololens, and Microsoft Visual Studio 2017. It visually displays the structure of virtual human organs to help doctors understand their conditions more clearly.

The article "Perioperative Nursing Care of Vascular Decompression for Trigeminal Neuralgia under AR Medical Technology" was retracted in 2022. Reason: concerns about the peer review.

#### 3.2.3. Acquisition of the Virtual Model

In medical diagnosis, two-dimensional images of the patient's organs can be collected with the help of professional medical equipment, and different two-dimensional images of the locations of interest of medical staff are obtained in different ways. For example, X-rays are used to collect projection images of bone tissue, and CT is used to collect tomographic data of brain tissue or internal organs, so as to observe and analyze the location to be diagnosed. Traditional doctor diagnosis only uses two-dimensional image data, and the diseased location and its internal structural information cannot be displayed directly in front of the doctor's eyes, which will interfere with the doctor's diagnosis and cause problems such as misdiagnosis. The three-dimensional visualization of the two-dimensional image data can observe all angles of the diseased location, thereby helping the doctor to observe the information of the lesion tissue more clearly. In this article, for head and face assisted surgery, the two-dimensional medical data used for modeling is the CT data in the tomographic image data.

The collected CT data is saved as a DICOM format file. It consists of three parts, namely, the introduction, the prefix, and the three-dimensional spatial data field (also called the data set). The first two are similar to the header of the file, including the description and format information of the image data. The single volume data element in the three-dimensional data field is in accordance with Arrange in a specific order. Here, we are most interested in the two-dimensional image data in the data field. There are two main methods of using the data field to reconstruct the three-dimensional structure of the model. One is to directly perform volume rendering, and the volume rendering directly uses the collected volume data for reconstruction.

This part of the experiment proposes that the above steps are used to carry out the perioperative nursing research experiment of vascular decompression for the treatment of trigeminal neuralgia under AR medical technology. The specific process is shown in Figure 2.

## 4. Experiment and Result Analysis

### 4.1. Perioperative Nursing Needs for Vascular Decompression in the Treatment of Trigeminal Neuralgia under AR Medical Technology

1. Follow up 100 patients by telephone or outpatient service. Through a questionnaire survey of 100 patients' operation-related conditions, 98 questionnaires were returned, with a recovery rate of 98%. Use the data from these questionnaires for the following analysis and research. Record and analyze the occurrence of surgery-related complications within one month after the surgery. According to the conclusions of relevant literature data, the main possible complications after surgery are hearing loss or tinnitus, facial paralysis or facial numbness, weakness in chewing, loss of taste, cerebrospinal fluid rhinorrhea, intracranial infection, aseptic meningitis, and Cestan-Chenais's Syndrome (ataxia, hypoesthesia, nystagmus, miosis, throat palsy). The incidence of postoperative complications of patients is shown in Table 2 and Figure 3.
2. The clinical incidence of trigeminal neuralgia is relatively high. The incidence rate of severe and mild cases in 100 patients is as high as 61%. The pathogenesis is relatively complicated. There is a lack of research on large clinical cases of the disease. Which surgical method is safer and effective is still worth studying.
3. The specific situation of the recurrence rate of the patients after three months, six months, one year, and two years after treatment is shown in Table 3 and Figure 4.
4. It can be seen from the figure that the patient's recurrence rate gradually decreased, but the recurrence rate increased slightly after two years, indicating that this technology can prevent patients from recurring in a short period of time, and it is ineffective for a long time. With the development of minimally invasive neurosurgery, microvascular decompression has been continuously improved and improved, and clinical treatment experience has been continuously enriched. Starting from the etiology of the disease, it has gradually replaced traditional surgical treatment methods. In the treatment of trigeminal neuralgia, microvascular decompression can effectively improve the effect of surgical treatment and reduce the occurrence of complications, and it is worthy of clinical application.
5. Investigate the patient's pain in the perioperative period, and plot the results into charts, as shown in Table 4 and Figure 5.

The article "Perioperative Nursing Care of Vascular Decompression for Trigeminal Neuralgia under AR Medical Technology" was retracted in 2022. Reason: concerns about the peer review.

Among the 100 patients surveyed, 46% of the patients felt mild pain before admission, 36% felt moderate pain before admission, and 12% felt severe pain; within 24 hours after receiving surgery 54% of patients said they felt mild pain, 37% of patients said there was no pain, and 9% of patients had moderate to severe pain; 72 hours after surgery, the vast majority of patients thought there was no pain, but 19% of them still felt no pain. The patient expressed pain.

Based on the above, it can be seen that careful perioperative care of patients is very necessary. In order to maintain the health and safety of patients, AR technology is applied to the perioperative care of vascular decompression for the treatment of trigeminal neuralgia; combined with advanced and intelligent technology, it is conducive to better care for patients and promote recovery.

### 4.2. Experiment Analysis

1. Use the algorithm of this paper to detect the three-dimensional medical human body model, etc., select five sets of the same samples for experiments under the two different conditions of light and darkness, and statistically organize the accuracy of related detection, as shown in Table 5 and Figure 6.
2. From the data in the chart, we can see that the average accuracy of the AR 3D detection algorithm in this paper is 96.6% under light conditions, and the average detection accuracy under dark conditions is 90.5%; the algorithm has better detection performance under light conditions.
3. After the patient receives perioperative care of vascular decompression for the treatment of trigeminal neuralgia under AR medical technology, a return visit will be made to the patient's feedback after receiving the nursing care improved by the new technology through the telephone or outpatient service, and the results collect statistics and draw graphs, as shown in Table 6 and Figure 7.

It can be clearly seen from the chart that the vast majority of patients believe that this type of care can help them recover faster, accounting for 96%; 94% of patients like this type of care; 88% of patients believe that this type of care is more humane. It can be seen that the perioperative care of vascular decompression for the treatment of trigeminal neuralgia under the AR medical technology proposed in this article has achieved initial success.

## 5. Conclusions

In recent years, due to the combination of computer application technology and medicine, the development of intersecting medical treatment has been continuously strengthened. Digital medical technology has gradually been adopted by hospitals at all levels. The current clinical surgery and nursing care are generally more precise, efficient, and safe. There are countless applications of AR technology in medicine, and with the continuous development of AR technology and the close integration of AR technology and medicine, AR medical technology has developed by leaps and bounds. This article proposes the application of AR technology to the perioperative nursing of vascular decompression surgery for trigeminal neuralgia and designs intelligent system architecture for the application of AR technology to the perioperative nursing of vascular decompression surgery for trigeminal neuralgia. Due to limited resources and its own capabilities, this research still has many shortcomings, such as insufficient experimental data and insufficient experimental samples. And it is difficult to master computer application technology in the research process. The research in this article is a combination of computers and nursing. It is hoped that it can promote the development of medical nursing and provide a foundation for the development of medical nursing in the future. It is believed that intelligent medical nursing will flourish in the future.

The article "Perioperative Nursing Care of Vascular Decompression for Trigeminal Neuralgia under AR Medical Technology" was retracted in 2022. Reason: concerns about the peer review.

## Figures and Tables

**Figure 1:** AR system.

**Figure 2:** Some steps of the experiment in this article.

**Figure 3:** Postoperative complications of the patient.

**Figure 4:** The patient's relapse after treatment.

**Figure 5:** Pain in patients during the perioperative period.

**Figure 6:** Detection accuracy.

**Figure 7:** Patient feedback.

**Table 1:** Part of the technical process of the method in this article.

Perioperative nursing research method of vascular decompression for trigeminal neuralgia under AR medical technology	2.1	Overview of trigeminal neuralgia	1	Symptom
			2	Treatment
	2.2	Perioperative nursing related research	1	Perioperative care
			2	Advantages of intelligent perioperative nursing
	2.3	AR medical technology related algorithms	1	Multisensor fusion algorithm
			2	Three-dimensional plane inspection
			3	Medical AR image segmentation

**Table 2:** Postoperative complications of patients.

Complication	Total number of patients	Number of patients	Percentage (%)
Hearing loss	100	12	12
Tinnitus	100	9	9
Facial paralysis	100	8	8
Weak chewing	100	11	11
Decreased taste	100	7	7
Cerebrospinal fluid rhinorrhea	100	2	2
Intracranial infection	100	5	5
Aseptic meningitis	100	6	6
Cestan-Chenais syndrome	100	1	1

**Table 3:** Recurrence of patients after treatment.

Time	Number of patients	Percentage (%)
Within three months	22	22
Within six months	19	19
Within one year	17	17
Within two years	21	21

**Table 4:** Pain in patients during the perioperative period.

Pain degree	Before admission (%)	24 hours after surgery (%)	72 hours after surgery (%)
No pain	3	37	81
Slight pain	46	54	15
Moderate pain	39	7	3
Severe pain	12	2	1

**Table 5:** Detection accuracy.

Detection accuracy	Bright (%)	Dark (%)
Sample 1	96.4	91.4
Sample 2	95.2	89.6
Sample 3	97.6	92.3
Sample 4	98.3	88.7
Sample 5	95.7	90.5
Average	96.6	90.5

**Table 6:** Patient feedback.

Serial number	Survey content	Yes	Yes-percentage (%)	No	No-percentage (%)
1	Do you like this kind of nursing?	94	94	6	6
2	Can this kind of nursing reduce your psychological burden?	87	87	13	13
3	Can this kind of care help you recover faster?	96	96	4	4
4	Is this kind of nursing more humanized?	88	88	12	12
5	Does this kind of care help you relieve pain?	81	81	19	19

The article "Perioperative Nursing Care of Vascular Decompression for Trigeminal Neuralgia under AR Medical Technology" was retracted in 2022. Reason: concerns about the peer review.

## Data Availability

Data sharing is not applicable to this article as no datasets were generated or analyzed during the current study.

## References

[1] Marchand E., Uchiyama H., Spindler F. (2016). Pose estimation for augmented reality: a hands-on survey. *IEEE Transactions on Visualization and Computer Graphics*.

[2] Matsutomo S., Manabe T., Cingoski V., Noguchi S. (2017). A computer aided education system based on AR by immersion to 3-D magnetic field. *IEEE Transactions on Magnetics*.

[3] Prasad S., Galetta S. (2016). Trigeminal neuralgia. *Neurologist*.

[4] Roesner F., Kohno T., Molnar D. (2016). Security and privacy for AR systems. *Communications of the ACM*.

[5] Cruccu G., Finnerup N. B., Jensen T. S. (2016). Trigeminal neuralgia. *Neurology*.

[6] Oliveira L. C. D., Soares A. B., Cardoso A., Andrade A. D. O., Lamounier Júnior E. A. (2016). Mobile augmented reality enhances indoor navigation for wheelchair users. *Research on Biomedical Engineering*.

[7] Lee Y.-H., Yin K., Wu S.-T. (2017). Reflective polarization volume gratings for high efficiency waveguide-coupling augmented reality displays. *Optics Express*.

[8] Sudana A. A. K. O., Aristamy I. G. A. A. M., Wirdiani N. K. A. (2016). Augmented reality application of sign language for deaf people in android based on smartphone. *International Journal of Software Engineering and Its Applications*.

[9] Borgmann H., Socarrás R., Salem J. (2017). Feasibility and safety of AR-assisted urological surgery using smartglass. *World Journal of Urology*.

[10] Farzeeha D., Omar M., Boon Y. (2018). The use of AR learning environment in enhancing students’ mental rotation skills. *Advanced Science Letters*.

[11] Mirauda D., Erra U., Agatiello R. (2018). Mobile AR for flood events management. *International Journal of Sustainable Development and Planning*.

[12] Zhang L., Chen S., Dong H., El Saddik A. (2018). Visualizing toronto city data with HoloLens: using augmented reality for a city model. *IEEE Consumer Electronics Magazine*.

[13] Jung T. H., Lee H., Chung N., tom Dieck M. C. (2018). Cross-cultural differences in adopting mobile augmented reality at cultural heritage tourism sites. *International Journal of Contemporary Hospitality Management*.

[14] Croatti A., Ricci A., Viroli M. (2017). Towards a mobile augmented reality system for emergency management. *International Journal of Distributed Systems and Technologies*.

[15] Cheng K.-H. (2017). Exploring parents’ conceptions of augmented reality learning and approaches to learning by augmented reality with their children. *Journal of Educational Computing Research*.

The article "Perioperative Nursing Care of Vascular Decompression for Trigeminal Neuralgia under AR Medical Technology" was retracted in 2022. Reason: concerns about the peer review.

[16] Louges M.-A., Kleiber J.-C., Bazin A., Chays A., Dubernard X. (2020). Efficacy of microsurgical vascular decompression in trigeminal neuralgia. *European Annals of Otorhinolaryngology, Head and Neck Diseases*.

[17] Sinha V. D., Khanuja J. S., Shekhawat J. (2020). Comparative evaluation of microscopic vascular decompression and endoscopic vascular decompression for trigeminal neuralgia: a clinical study. *IP Indian Journal of Neurosciences*.

[18] Dou N.-N., Zhong J., Liu M.-X. (2016). Teflon might be a factor accounting for a failed microvascular decompression in hemifacial spasm: a technical note. *Stereotactic and Functional Neurosurgery*.

[19] Raghavendra H., Varsha K. S., Sobti S. (2019). Micro vascular decompression for trigeminal neuralgia: preliminary experience. *Journal of Medical and Scientific Research*.

[20] Kohshi K., Morimatsu Y., Morimatsu Y. (2017). Cerebrospinal vascular diseases misdiagnosed as decompression illness: the importance of considering other neurological diagnoses. *Undersea and Hyperbaric Medicine*.

[21] Dapena J. C., Lansdorp C. A., Lansdorp C. A., Mitchell S. J. (2020). Persistent extravascular bubbles on radiologic imaging after recompression treatment for decompression sickness: a case report. *Diving and Hyperbaric Medicine Journal*.

[22] Kang I. H., Park B. J., Park C. K., Malla H. P., Lee S. H., Rhee B. A. (2016). A clinical analysis of secondary surgery in trigeminal neuralgia patients who failed prior treatment. *Journal of Korean Neurosurgical Society*.

[23] Muratorio F., Tringali G., Levi V., Ligarotti G. K., Nazzi V., Franzini A. A. (2016). Hydrocephalus: an underrated long-term complication of microvascular decompression for trigeminal neuralgia. A single institute experience. *Acta Neurochirurgica*.

[24] Shibao S., Toda M., Yoshida K. (2016). Laser speckle imaging to improve clinical outcomes for patients with trigeminal neuralgia undergoing radiofrequency thermocoagulation response. *Journal of Neurosurgery*.

[25] Desebbe O., Lanz T., Kain Z., Cannesson M. (2016). The perioperative surgical home: an innovative, patient-centred and cost-effective perioperative care model. *Anaesthesia Critical Care & Pain Medicine*.

[26] Page A. J., Gani F., Crowley K. T. (2016). Patient outcomes and provider perceptions following implementation of a standardized perioperative care pathway for open liver resection. *British Journal of Surgery*.

[27] Aviles C., Hockenberry M., Vrochides D. (2017). Perioperative care implementation: evidence-based practice for patients with pancreaticoduodenectomy using the enhanced recovery after surgery guidelines. *Clinical Journal of Oncology Nursing*.

The article "Perioperative Nursing Care of Vascular Decompression for Trigeminal Neuralgia under AR Medical Technology" was retracted in 2022. Reason: concerns about the peer review.

[28] Fleming I. O., Garratt C., Guha R. (2016). Aggregation of marginal gains in cardiac surgery: feasibility of a perioperative care bundle for enhanced recovery in cardiac surgical patients. *Journal of Cardiothoracic and Vascular Anesthesia*.

[29] Watanabe M., Mine S., Nishida K. (2016). Improvement in short-term outcomes after esophagectomy with a multidisciplinary perioperative care team. *Esophagus*.

[30] Allana A., Mujtaba N. (2020). Perioperative care of the pregnant patient undergoing non-obstetric surgery. *British Journal of Hospital Medicine (London, England: 2005)*.

